The article "Automatic Detection of Coronary Metallic Stent Struts Based on YOLOv3 and R-FCN" was published in 2020. Journal: Comput Math Methods Med.

# Automatic Detection of Coronary Metallic Stent Struts Based on YOLOv3 and R-FCN

**DOI:** 10.1155/2020/1793517

**Published:** 2020-09-01

**Authors:** Xiaolu Jiang, Yanqiu Zeng, Shixiao Xiao, Shaojie He, Caizhi Ye, Yu Qi, Jiangsheng Zhao, Dezhi Wei, Muhua Hu, Fei Chen

**Affiliations:** ^1^Chengyi University College, Jimei University, Xiamen 361021, China; ^2^School of Informatics, Xiamen University, Xiamen 361021, China; ^3^School of Management, Xiamen University, Xiamen 361021, China; ^4^School of Mathematical Sciences, Xiamen University, Xiamen 361021, China; ^5^Department of Cardiology, Tongji Hospital of Tongji University, Shanghai 200065, China

## Abstract

An artificial stent implantation is one of the most effective ways to treat coronary artery diseases. It is vital in vascular medical imaging, such as intravascular optical coherence tomography (IVOCT), to be able to track the position of stents in blood vessels effectively. We trained two models, the “You Only Look Once” version 3 (YOLOv3) and the Region-based Fully Convolutional Network (R-FCN), to detect metal support struts in IVOCT, respectively. After rotating the original images in the training set for data augmentation, and modifying the scale of the conventional anchor box in both two algorithms to fit the size of the target strut, YOLOv3 and R-FCN achieved precision, recall, and AP all above 95% in 0.4 IoU threshold. And R-FCN performs better than YOLOv3 in all relevant indicators.

## 1. Introduction

Coronary artery disease (CAD) is one of the most frequent causes of death despite being treatable. For treating the obstructive plaques, stenting is commonly used of the bare metal stent (BMS), the drug-eluting stent (DES), or bioresorbable vascular scaffolds (BVS). After implantation, the stents have to be assessed to detect malposition or endothelialisation. Intravascular optical coherence tomography (IVOCT) is one of imaging modality with the resolution and contrast necessary to enable accurate measurements of luminal architecture and neointima stent coverage.  Figure 1 shows an IVOCT image frame after metallic stent implantation. However, since a pullback of the IVOCT image sequence for a single patient often contains hundreds of images and thousands of struts, it is labour-intensive and time-consuming to conduct a quantitative evaluation for every patient manually. Therefore, a fully automatic method for metallic strut analysis is highly desired. Until now, several different strategies [1–19] have been proposed for the detection of stent strut candidates in IVOCT and the removal of false positives.

Since metallic struts appear as high-reflecting spots followed by trailing shadows in IVOCT images, as shown in Figure 1, most algorithms are searching for these features to detect stent struts [1]. Lu et al. [2] trained a bagged decision tree classifier, using specific features extracted from the images to classify the candidate stent struts. Han et al. [3] applied the Laplacian filter to the image in the polar coordinates map to extract corners and edges and then used the intensity threshold to identify the stent struts. Nam et al. [4] detected the candidate struts by IVOCT intensity image and gradient image, and then by using a hidden layer and a ten-node artificial neural network determines the candidate struts. Migliori et al. [5] classified pixels associated with high slopes as candidate struts and applied a penalty function away from the lumen contour structure.

Alternative approaches for stent strut detection as follow. A controllable filter is designed by Xu et al. [6] to calculate the local ridge strength and direction to locate the deeply buried struts. Wang et al. [7] used the Bayesian network and the stent mesh information of the adjacent frame to determine the location of the struts in the A-scan. They used the graph cut algorithm to simultaneously locate the exact struts depth positions in the IVOCT pullback.

In recent years, a deep learning framework has achieved excellent results in the computer visual object detection and recognition domain, and it has attracted increasing attention and led to more research based on this framework. Traditional machine learning methods depend on manually designed features. Unlike that, novel representation patterns or models are automatically learned from low-level features to high-level semantics in deep learning, which often makes the detection performance more correct and robust. BVS detection in IVOCT images based on deep learning has been reported recently. Cao et al. [8] constructed a region-based fully convolutional network (R-FCN) detector for BVS detection in IVOCT images. Zhou et al. [9] proposed an automatic detection method for BVS based on a U-shaped convolutional neural network. Gessert et al. [10] can predict whether image slices contain metal supports, BVS, or do not contain any equipment only using image-level tags by a trained convolutional neural network, achieving 99.0% classification accuracy. However, there are few methods for detecting metallic stents based on deep learning. Given this, in this paper, we attempt to use two deep learning object detection models to detect metallic stents and compare the performance.

Conventional deep learning models for object detection fall into two types: one-stage and two-stage. YOLOv3 and R-FCN are, respectively, typical algorithms of these two types, and also are frequently used in the medical field. Wu et al. [11] developed a deep learning model (BMSNet) with the YOLOv3 architecture for assisting haematologists in the interpretation of bone marrow smears for faster diagnosis and disease monitoring. Park et al. [12] compared the performance of various state-of-the-art deep-learning architectures, including YOLOv3, for detecting the optic nerve head and vertical cup-to-disc ratio in fundus images. Safdar et al. [13] highlighted the most suitable Data Augmentation technique for medical imaging by using YOLOv3. Wu et al. [14] investigated the potential for using Principal Component Analysis (PVA) and Adaptive Median Filter (AMF) to improve four algorithms, including R-FCN and YOLOv3. Zhang et al. [15] proposed a novel abnormal region detection approach for cervical screening based on R-FCN. Morrell et al. [16] presented a neural net architecture based on R-FCN to suit mammograms.

Since YOLOv3 and R-FCN perform well in medical fields, we used them in this paper for metallic stent struts detection and tried to compare the performance of these two models systematically. We also realised the data augmentation of the existing training set through images rotation to enhance the advantage of big data in feature extraction. To explore the use of anchor box in specialized fields, we also adjusted its size to suit the detection of metallic stent struts: *k*-means clustering in YOLOv3, manually fixed in R-FCN.

## 2. Material and Methods

### 2.1. Dataset

For validating the algorithm, ten pull-back runs were acquired with an IVOCT imaging system from a baseline study. The pull-back speed was 15 mm/s. All of the stents were metallic stents. The total stent length was 21 2.17 mm. The different patients who participated in the study were independent of each other. As shown in Figure 1, the IVOCT image contains the stent, guidewire, imaging catheter, protective sheath, blood artefacts, and lumen border. To assist medical personnel in judging the location and performance of the stent, we need to identify the metallic stent in these complex backgrounds automatically. There are 165 IVOCT images, and each image has about 3∽22 metallic stent struts, which has manually marked all the stent struts as the ground truth by rectangular frames.

### 2.2. Deep Learning Object Detection Model

There are two types of deep learning models for object detection: one-stage and two-stage. Two-stage object detection strategy consists of: (i) region proposal, and (ii) region classification. Typical two-stage model includes R-CNN [20], Fast R-CNN [21], Faster R-CNN [22], and R-FCN [23]. The one-stage model is an end-to-end algorithm. It does not need to generate candidate frames and directly transform the problem of object frames positioning into a regression problem. The typical 1-stage model includes the YOLO series [24–26] and SSD [27]. Generally speaking, the method based on candidate regions has higher accuracy, but the end-to-end way has distinct advantages in speed. In this paper, R-FCN and YOLOv3 are compared, and they are used to detect the metallic stent struts in the IVOCT image.

### 2.3. YOLOv3

Given the input image, YOLOv1 directly returns the object's bounding box and its category at multiple locations in the image. YOLOv2 and YOLO9000 introduced anchor boxes to predict the offset and confidence of the anchor boxes instead of directly predicting the coordinate values. By adding a pass-through layer, the high-resolution shallow features are connected to the low-resolution features for fusion and detection. YOLOv3 detects objects on multiple fusion feature maps separately, which improves efficiency in the detection of smaller objects. At the same time, the classification uses multiple logistic classifiers instead of a softmax classifier, which is used to solve the multilabel classification problem in YOLOv2.

#### 2.3.1. Overall Architecture of YOLOv3

The network architecture of YOLOv3 (Figure 2) is divided into three parts: darknet53 for feature extraction, YOLO layers for feature fusion, and classification and location. Darknet53 has a total of 53 convolutional layers, and the rest are residual layers. The YOLO layers are used for feature fusion to generate three scale feature maps. It takes feature maps from earlier in the network and merges it with the upsampled features using concatenation. Object classification and locating are carried out on the feature fusion maps of three scales (13∗13, 26∗26, or 52∗52), respectively, to the different size objects for detection.

#### 2.3.2. Unified Detection of YOLOv3

Taking the 13∗13 fusion feature map as an example, YOLOv3 divides the map into 13∗13 grids. If the center of an object falls into a grid cell, the grid cell is responsible for detecting the object. Each grid cell predicts three bounding boxes, thus, returning 3∗(4 + 1 + C) tensors, of which four bounding box offsets, one confidence score, and C conditional class probabilities. Four bounding box offsets refer to the offsets from the given anchor box. Each scale needs three anchor boxes as bounding boxes prior, so a total of 9 anchor boxes are clustered from our data set before. Including all cells, the scale feature map outputs 13∗13∗3∗(5 + C) tensors. Adding the output of 26∗26 and 52∗52 scale feature maps, we get a total of (13∗13 + 26∗26 + 52∗52)∗3∗(5 + C) tensor.

As shown in Figure 3, the four bounding box offsets *t*_*x*_, *t*_*y*_, *t*_*w*_, *t*_*h*_ can be converted into the center coordinates *b*_*x*_, *b*_*y*_ and the width *b*_*w*_ and the height *b*_*h*_ of the bounding box by formula:

(1) $$\begin{array}{c} b_{x}=\sigma \left(t_{x}\right)+c_{x}, \end{array}$$

(2) $$\begin{array}{c} b_{y}=\sigma \left(t_{y}\right)+c_{y}, \end{array}$$

(3) $$\begin{array}{c} b_{w}=p_{w}e^{t_{w}}, \end{array}$$

(4) $$\begin{array}{c} b_{h}=p_{h}e^{t_{h}}, \end{array}$$

where *P*_*w*_ and *P*_*h*_ are the width and height of the prior box, *C*_*x*_ and *C*_*y*_ are the offsets of the responsible grid from the upper left corner of the image, and *σ* is the sigmoid function.

The objectness score reflects the confidence that the grid cell contains objects and the accuracy of predicting that the cell contains objects,

(5) $$\begin{array}{c} \text{objectness score}=\mathrm{Pr}\left(\text{object}\right)\times {\text{IoU}}_{\text{pred}}^{\text{truth}}. \end{array}$$

When there are objects in the cell, the objectness score will be equal to the intersection over union (IoU) between the bounding box and the ground truth:

(6) $$\begin{array}{c} {\text{IoU}}_{\text{pred}}^{\text{truth}}=\frac{\text{ground truth box}\cap \text{predicted bounding box}}{\text{ground truth box}\cup \text{predicted bounding box}}. \end{array}$$

C conditional class probabilities Pr(class_*i*_|object) are conditioned on the grid cell containing an object. The final category of confidence is

(7) $$\begin{array}{c} \mathrm{Pr}\left({\text{class}}_{i}\left|\text{object}\right.\right)\times \mathrm{Pr}\left(\text{object}\right)\times {\text{IoU}}_{\text{pred}}^{\text{truth}}=\mathrm{Pr}\left({\text{class}}_{i}\right)\times {\text{IoU}}_{\text{pred}}^{\text{truth}}. \end{array}$$

#### 2.3.3. Training YOLOv3

The final loss function will summarize the losses of the three scales. During training, the error function of each scale includes a localization error, a confidence error, and a classification error. Using the formula (1)–(4) to inverse the four coordinates ${\hat{x}}_{i},{\hat{y}}_{i},{\hat{w}}_{i},{\hat{h}}_{i}$ corresponding to the ground truth in cell *i*, we can calculate SSE of the corresponding predicted coordinates *x*_*i*_, *y*_*i*_, *w*_*i*_, *h*_*i*_ as the localization error. YOLOv3 uses logistic regression to predict the confidence score *c*_*i*_, and the actual score ${\hat{c}}_{i}$ is depending on the IoU of the bounding box prior and ground truth. Then, the binary cross-entropy of the predicted and actual confidence score is the confidence loss. YOLOv3 uses independent logistics instead of softmax as the classifier. For each category, binary cross-entropy is also used as the loss function. Two parameters *λ*_coord_ and *λ*_noobj_ can adjust the balance of the loss from bounding box coordinate predictions and the loss from confidence predictions for boxes that do not contain objects. The final loss a function is

(8) $$\begin{array}{c} \text{Loss}={\text{Error}}_{\text{localization}}+{\text{Error}}_{\text{confidence}}+{\text{Error}}_{\text{class}},\\ {\text{Error}}_{\text{localization}}=\lambda_{\text{coord}}\overset{S^{2}}{\underset{i=0}{\sum }}\overset{B}{\underset{j=0}{\sum }}I_{ij}^{\text{obj}}\left[{\left(x_{i}-{\hat{x}}_{i}\right)}^{2}+{\left(y_{i}-{\hat{y}}_{i}\right)}^{2}\right]+\lambda_{\text{coord}}\overset{S^{2}}{\underset{i=0}{\sum }}\overset{B}{\underset{j=0}{\sum }}I_{ij}^{\text{obj}}\left(2-w_{i}\times h_{i}\right)\left[{\left(w_{i}-{\hat{w}}_{i}\right)}^{2}+{\left(h_{i}-{\hat{h}}_{i}\right)}^{2}\right],\\ {\text{Error}}_{\text{confidence}}=-\overset{S^{2}}{\underset{i=0}{\sum }}\overset{B}{\underset{j=0}{\sum }}I_{ij}^{\text{obj}}\times \left[{\hat{c}}_{i}\times \log c_{i}+\left(1-{\hat{c}}_{i}\right)\times \log\left(1-c_{i}\right)\right]-\lambda_{\text{noobj}}\overset{S^{2}}{\underset{i=0}{\sum }}\overset{B}{\underset{j=0}{\sum }}I_{ij}^{\text{noobj}}\times \left[{\hat{c}}_{i}\times \log c_{i}+\left(1-{\hat{c}}_{i}\right)\times \log\left(1-c_{i}\right)\right],\\ {\text{Error}}_{\text{class}}=-\overset{S^{2}}{\underset{i=0}{\sum }}I_{i}^{\text{obj}}\underset{c\in \text{classes}}{\sum }\left[{\hat{p}}_{i}\left(c\right)\times \log p_{i}\left(c\right)+\left(1-{\hat{p}}_{i}\left(c\right)\right)\times \log\left(1-p_{i}\left(c\right)\right)\right], \end{array}$$

where *S*^2^ is the number of grid cells, *B* is the number of anchor boxes. By minimizing the loss function to learn the weights, we can obtain the location of the bounding box and the category prediction.

### 2.4. Region-Based Fully Convolutional Networks (R-FCN)

R-FCN is a typical two-stage object detection method. In the first stage, the Regional Proposal Network (RPN) is used for regional proposals to generate candidate RoI. In the second stage, R-FCN uses position-sensitive score maps to synthesize the features of different positions of ROIs so that the network can solve the dilemma between the translation invariance in classification and the translation variance in object detection. At the same time, all the learnable weight layers are convolutional and can be calculated in the whole image. Finally, the entire network reaches the structure of full convolution, which significantly improves efficiency.

#### 2.4.1. Overall Architecture of R-FCN

The overall architecture of the metallic stent strut detection based on R-FCN is shown in Figure 4. After extracting features through a series of convolutions in Resnet-50, a Region Proposal Network (RPN) uses a small sliding window and anchor boxes to generate candidate regions on a whole feature map. For the metallic stent strut and the background, the feature map of the entire image is, respectively, connected with 3∗3 position-sensitive score maps by convolution. Combining the RoI pooling of 9 position-sensitive scores, the category probability corresponding to each RoI can be voted. The four localization parameters that represent the offset from the anchor boxes are also obtained by voting similarly. After training the network, R-FCN outputs the adjusted new position and score of the metallic stent strut RoIs as “R-FCN output.” If the category score of each RoI is less than the score threshold, we remove the bounding box to get a “Threshold output.” The remaining bounding boxes still have a lot of overlap. Run a nonmaximum suppression (NMS), and only the bounding box with the highest score is kept where the IoU exceeds a certain threshold. The remaining bounding box is the final “Detection result.”

#### 2.4.2. Region Proposal Network (RPN)

RPN uses a fully convolutional network to output a set of rectangular region proposals at once on the entire feature map. Slide a small sliding window on the feature map, and use each area located by it as input. If *k* (*k* = 9) anchor boxes are used as the regression reference, each sliding window will output 4 k coordinate regression *t*_*x*_, *t*_*y*_, *t*_*w*_, *t*_*h*_ and 2 k bounding box classification to estimate the probability that each proposal is the object or not.

The RPN loss function consists of two parts, the log classification loss, and the smooth regression loss:

(9) $$\begin{array}{c} \begin{array}{c} L\left(\left\{p_{i}\right\},\left\{t_{i}\right\}\right)=\frac{1}{N_{cls}}\underset{i}{\sum }L_{cls}\left(p_{i},p_{i}^{*}\right)+\lambda \frac{1}{N_{\text{reg}}}\underset{i}{\sum }p_{i}^{*}L_{\text{reg}}\left(t_{i},t_{i}^{*}\right),\\ L_{cls}\left(p_{i},p_{i}^{*}\right)=-p_{i}^{*}\times \log p_{i}-\left(1-p_{i}^{*}\right)\times \log\left(1-p_{i}\right),\\ L_{\text{reg}}\left(t_{i},t_{i}^{*}\right)={\text{smooth}}_{L_{1}}\left(t_{x}-t_{x}^{*}\right)+{\text{smooth}}_{L_{1}}\left(t_{y}-t_{y}^{*}\right)+{\text{smooth}}_{L_{1}}\left(t_{w}-t_{w}^{*}\right)+{\text{smooth}}_{L_{1}}\left(t_{h}-t_{h}^{*}\right), \end{array} \end{array}$$

where the smooth *L*_1_ is defined by

(10) $$\begin{array}{c} {\text{smooth}}_{L_{1}}\left(x\right)=\left\{\begin{array}{cc} 0.5x^{2} & \text{if }\left|x\right|<1,\\ \left|x\right|-0.5 & \text{otherwise}, \end{array}\right. \end{array}$$

{*p*_*i*_}, {*t*_*i*_} are the outputs of the anchor in the classification layer and regression layer. During training, we assign labels to the anchor based on the IoU of the anchor *i* and the ground truth box. A positive label is 1, and a negative label is 0. *t*_*i*_^∗^ is the vector about the ground truth box location associated with the positive anchor.

RPN only relies on a single-scale image and feature mapping, uses a single-size filter, and thus generates a region proposal that is translation-invariant. Shared features require no additional cost to process the scale of the object.

#### 2.4.3. Position-Sensitive Score Maps

The innovation of R-FCN is the position-sensitive score map. Object classification and location all need 3∗3 score maps. We take the position-sensitive score maps of the stent strut classification as an example. 9 position-sensitive score maps correspond to features of nine positions of the strut. Each position-sensitive map in the RoI area is divided into 3∗3 bins, and a position-sensitive RoI pooling operated only over the appropriate bin of each score map:

(11) $$\begin{array}{c} r_{c}\left(i,j\left|\Theta \right.\right)=\underset{\left(x,y\right)\in \text{bin}\left(i,j\right)}{\sum }z_{i,j,c}\left(x+x_{0},y+y_{0}\left|\Theta \right.\right)/n. \end{array}$$

Nine pool responses vote on the RoI by averaging; then, the classification probability of RoI is output by the softmax function.

(12) $$\begin{array}{c} r_{c}\left(\Theta \right)=\underset{i,j}{\sum }r_{c}\left(i,j\left|\Theta \right.\right),\\ s_{c}\left(\Theta \right)=e^{r_{c}\left(\Theta \right)}/\overset{C}{\underset{c^{\prime }=0}{\sum }}e^{r_{c^{\prime }}\left(\Theta \right)}. \end{array}$$

Bounding box regression is similar, except that the output after voting is the 4 d vector (*t*_*x*_, *t*_*y*_, *t*_*w*_, *t*_*h*_).

The loss function for each RoI includes cross-entropy loss for classification and regression loss for the location of the positive sample:

(13) $$\begin{array}{c} L\left(s,t_{x,y,w,h}\right)=L_{cls}\left(s_{c^{*}}\right)+\lambda \left[C^{*}>0\right]L_{\text{reg}}\left(t,t^{*}\right),\\ L_{cls}\left(s_{c^{*}}\right)=-s_{c^{*}}\times \log s-\left(1-s_{c^{*}}\right)\times \log\left(1-s\right). \end{array}$$

Regression loss is the same as RPN's. *C*^∗^ represents the label of the RoI. [*C*^∗^ > 0] means that if the label is positive, it is equal to 1; otherwise, it is 0.

### 2.5. Performance Measures

precision (P), recall (R), and AP are principal quantitative indicators for algorithm performance evaluation in deep learning, which are employed in this experiment.

Denote by *TP*, *FP*, and *FN* the numbers of true positives, false positives, and false negatives, respectively. Then, precision and recall are computed as follows:

(14) $$\begin{array}{c} \text{Precision }=\;\frac{\text{TP}}{\text{TP}+\text{FP}},\\ \text{Recall }=\;\frac{\text{TP}}{\text{TP}+\text{FN}}. \end{array}$$

Here, whether a bounding box belongs to TP or FP depends on the IoU threshold of the ground truth and bounding box.

Here, AP refers to the average precision, the area under the P-R curve by numerical integration. The computation of it is shown as follows:

(15) $$\begin{array}{c} \text{AP }=\;\underset{n}{\sum }\left(R_{n}-R_{n-1}\right)P_{n}, \end{array}$$

where *P*_*n*_ and *R*_*n*_ are the precision and recall at the nth threshold.

## 3. Results and Discussion

### 3.1. Data Preprocessing

To effectively detect the metallic stent strut, we cropped the extraneous edges in all the IVOCT images, so that the image size changes from 704∗704 to 450∗450. Of all 165 IVOCT images, we used 100 images as the training set, 33 images as the verification set for adjusting hyperparameters, and 32 images as the test set. To augment the training of samples, we rotated the training set images. Along the catheter centre, a new training set image is generated every 30 degrees of rotation, and finally, 1200 images are obtained as the training set (Figure 5).

### 3.2. Parameters Setting

Only one type of metallic stent strut is to be detected. We take C the number of categories in YOLOv3 and R-FCN as 1. Due to the relatively small size of the stent struts, the anchor box should be different from the usual. Through the *K*-means algorithm, nine anchor boxes were clustered in YOLOv3 with the data set, which size results in 12 × 14, 14 × 18, 15 × 15, 18 × 18, 19 × 26, 19 × 15, 24 × 19, 29 × 26, 30 × 16. As a comparison, the anchor boxes in R-FCN is manually fixed to the length of {8, 16, 32} and the ratio of {0.85, 1, 1.85}.

In YOLOv3, we set 0.1 as the IoU threshold to mark positive labels, and the threshold in the objectiveness score is also set to 0.1. The coordinate weight *λ*_coord_ and the no object weight *λ*_noobj_ in the loss function adopt the default values of 5 and 0.5.

In R-FCN, the positive overlap in RPN has a threshold of 0.7, while the threshold in “R-FCN output” is 0.1, and in NMS, it is 0.3.

### 3.3. Results and Discussion

The test results are shown in Table 1. We compared the performance of YOLOv3 and R-FCN corresponding to different IoU between the bounding box and the ground truth. As the IoU threshold gradually increases, the precision, recall, and AP decrease slowly in both algorithms. When the IoU threshold is less than 0.45, all the indicators are above 92.7%. When 0.4 IoU threshold, they even all reach above 95%. And it is not hard to find that the R-FCN is superior to the YOLOv3 for any of the IoU thresholds.

Table 1 shows that the difference between YOLOv3 and R-FCN in precision is higher than that in the recall. It indicates that false positives (FP) are more likely to occur in YOLOv3 than false negatives (FN). For example, when the IoU threshold is 0.4, the number of false positives based on R-FCN is only 2, but yolov3 reaches 15. The difference between the two methods in the recall is only 0.2%, but in precision is 3.1%.

Examples of metallic stents detecting results got by YOLOv3 and R-FCN in the same image sets show more comparison in Figures 6 and 7 (when IoU = 0.4). The green dashed boxes refer to the ground truth, and those in red refer to bounding boxes in both figures. The boxes which are pointed at by the white arrow in Figure 7 refer to false positives, while those by yellow arrow refer to false negatives.  Figure 6 shows that both algorithms perform quite well in metallic stents detection. But it is easy to find that YOLOv3 has some false positives while R-FCN does not have in the same image sets in Figure 7. R-FCN has better performance in samples with unobvious characteristics, most of which are located in the areas where the color changes or the stent struts are denser.

In general, both of YOLOv3 and R-FCN algorithms performed pretty well in metallic stents detection (Figure 6(a)–6(c) and Figures 6(d)–6(f)). However, R-FCN has better performance in obscure samples, such as images with intimal hyperplasia or noise interference (Figures 7(a)–7(c) and Figures 7(d)–7(f)).

## 4. Conclusion

In this paper, we presented two automatic methods for metallic stents detection based on YOLOv3 (one-stage) and R-FCN (two-stage), respectively. To augment the data, we rotated the images of the training data set. And we adjusted the size of the anchor box to adapt to the detection of small objects. The experiments demonstrate that both algorithms perform fairly well whether the characteristic of metallic stents is clear or blurred (on account of intimal hyperplasia and noise interference). When the IoU threshold of the ground truth and bounding box is set to 0.4, precision, recall, and AP all reach above 95%. Nevertheless, R-FCN performs better than YOLOv3 in all relevant indicators, as shown in Table 1. The precision of R-FCN reaches more than 99.3% when the IoU threshold is less than or equal to 0.45. The future work will mainly focus on adding the complexity of the network, combining multiple algorithms for reinforcement learning to improve the performance further.

## Figures and Tables

**Figure 1:** IVOCT image after metallic stent implantation.

**Figure 2:** Architecture of metallic stent detection based on YOLOv3.

**Figure 3:** Bounding boxes with dimension priors and location prediction.

**Figure 4:** Architecture of metallic stent detection based on R-FCN.

**Figure 5:** Data preprocessing.

**Figure 6:** Examples of metallic stents detection results by YOLOv3 (a–c) orc by R-FCN (d–f). The green dashed boxes refer to the ground truth, and those in red refer to bounding boxes (when IoU threshold = 0.4).

**Figure 7:** Examples of metallic stents detection result by YOLOv3 (a–c) or by R-FCN (d–f). The boxes which are pointed at by white arrow and yellow arrow refer to false positives and false negatives, respectively.

**Table 1:** Comparisons between R-FCN and YOLOv3 algorithms corresponding to various IoU threshold. The amount of stents for testing is 425.

IoU	TP		FP		Precision		Recall		AP	
	R-FCN	YOLOv3	R-FCN	YOLOv3	R-FCN	YOLOv3	R-FCN	YOLOv3	R-FCN	YOLOv3
0.30	409	410	1	12	99.8%	97.2%	96.2%	96.5%	96.2%	96.0%
0.35	408	409	2	13	99.5%	96.9%	96.0%	96.2%	96.0%	95.5%
0.40	408	407	2	15	99.5%	96.4%	96.0%	95.8%	96.0%	95.0%
0.45	407	402	3	20	99.3%	95.3%	95.8%	94.6%	95.7%	92.7%
0.50	403	391	7	31	98.3%	92.7%	94.8%	92.0%	94.2%	88.7%
0.55	386	376	24	46	94.1%	89.1%	90.8%	88.5%	88.4%	81.9%
0.60	353	347	57	75	86.1%	82.2%	83.1%	81.6%	76.5%	69.6%

## Data Availability

The data used to support the findings of this study are available from the corresponding author upon request.
